RETRACTED

# MiR-579 Inhibits Lung Adenocarcinoma Cell Proliferation and Metastasis via Binding to CRABP2

**DOI:** 10.1155/2022/9111681

**Published:** 2022-08-04

**Authors:** Qijun Yi, Yu'e Miao, Ying Kong, Yan Xu, Jinghao Zhou, Qi Dong, Haiyan Liu

**Affiliations:** Department of Chemotherapy, The Second Affiliated Hospital of Shandong First Medical University, Tai'an City, Shandong, China

## Abstract

**Background:**

Lung cancer is the cancer with the highest morbidity and mortality. Lung adenocarcinoma (LUAD) is a subtype of lung cancer. The aim of this study is to explore the functions of miR-579 and CRABP2 in lung adenocarcinoma.

**Methods:**

Cell counting kit-8 (CCK-8) and colony formation assays were applied to calculate cell proliferative abilities. Transwell assay was utilized to measure cell invasive ability.

**Results:**

MiR-579 is low expressed in LUAD tissues and cell lines. MiR-579 inhibits cell viability and invasion of lung adenocarcinoma. Knockdown of CRABP2 inhibits cell proliferation and invasion of Calu-3 cells. MiR-579 suppresses cell proliferation and invasion by regulating CRABP2 in Calu-3 cells.

**Conclusion:**

Our study reveals that miR-579 acts as a tumor suppressor in LUAD and miR-579 can target and regulate the expression of CRABP2 to mediate cell proliferation and invasion. This study indicates that miR-579 has a potential to be a candidate biomarker for the treatment of LUAD.

## 1. Introduction

Lung cancer is a health killer with high incidence, and its mortality rate ranks first among all cancers for many years [1]. Lung adenocarcinoma (LUAD) is a kind of non-small cell lung cancer, which is a subtype of lung cancer [2]. Despite advances in the diagnosis and treatment of lung cancer, the prognosis of patients remains poor with a 5-year survival rate less than 16% [3]. The lack of understanding of the biological mechanisms associated with LUAD limits the efficacy of treating LUAD. Due to the lack of effective diagnostic biomarkers, patients with LUAD are mainly diagnosed at an advanced stage. Therefore, it is crucial to explore the pathogenesis mechanism of LUAD to improve clinical efficacy.

microRNAs (miRNAs) are a class of conserved, small non-coding RNAs with 19 to 25 nucleotide that regulate developmental and physiological processes [4]. MiRNAs usually negatively regulate gene expression in a post-transcriptional manner by degrading mRNA or inhibiting translation [5, 6]. Accumulating evidences suggest that dysregulation of miRNAs frequently occurs during lung adenocarcinoma initiation [7]. For instance, miRNA-885 inhibits docetaxel chemoresistance in lung adenocarcinoma by downregulating Aurora A [8]. MiR-22 is downregulated in lung adenocarcinoma and may serve as a biomarker for the diagnosis and prognosis of lung adenocarcinoma [9]. MiR-19b promotes lung adenocarcinoma metastasis via Hippo pathway [10]. These works strongly suggest a role of miRNAs in control of LUAD. It has been reported that miR-579 was expressed in non-small lung cancer [11]. However, the functions of miR-579 in lung adenocarcinoma are still unclear.

RETRACTED

Cellular retinoic acid binding protein 2 (CRABP2), a cytosol-to-nuclear shuttling protein, encodes a member of the retinoic acid, which binds protein family and lipocalin/cytosolic fatty-acid binding protein family [12]. CRABP2 is a cytosol-to-nuclear shuttling protein, which facilitates RA binding to its cognate receptor complex and transfer to the nucleus. CRABP2 is found to be upregulated in thyroid carcinoma and promoted the invasion, migration, and EMT of THCA cells [13]. Downregulation of CRABP2 inhibits proliferation and metastasis and promotes cell apoptosis of hepatocellular carcinoma [14]. This work reveals that miR-579 targets CRABP2 to regulate the biological process of lung adenocarcinoma and provides a research direction for the targeted therapy of LUAD.

## 2. Material and Methods

### 2.1. Sample Collection

During January 2012 to December 2018, 57 lung adenocarcinoma patients were collected from our hospital, and we obtained 57 pairs of LUAD tissue samples and corresponding paracancerous tissue samples through surgical operation. After surgical resection, all the tissues were rapidly frozen in liquid nitrogen and stored at − 80 °C. All the informed consents were obtained before this study, and the scheme was approved by the Ethics Committee of The Second Affiliated Hospital of Shandong First Medical University.

### 2.2. Cell Culture

Human LUAD cells (H1650, A549, and Calu-3) and a normal cell BEAS-2B were purchased from BeNa Culture Collection (Suzhou, Jiangsu, China). All the cells were cultured in Roswell Park Memorial Institute (RPMI)-1640 (Thermo Fisher Scientific Company, Waltham, Massachusetts, USA) supplemented with 10% fetal bovine serum (FBS; Hyclone, Logan, UT) at 37 °C.

### 2.3. Cell Transfection

MiR-579 mimic, miR-579 inhibitor, pcDNA3.1-CRABP2, si-CRABP2, and control were synthesized and purchased from GenePharma (Shanghai, China). Calu-3 cells were seeded in 6-well plat and cultured to the confluence of 70%. Cells were transfected using the Lipofectamine 2000 kit (Invitrogen, Carlsbad, CA, USA). Lipofectamine 2000 and serum-free medium were mixed and placed in a sterile Eppendorf (EP) tube for 5 minutes. Meanwhile, mix the vector and serum-free medium into another sterile EP tube. The solution in the above two test tubes was mixed and allowed to stand at room temperature for 20 minutes to obtain a complex of RNA and liposomes. This mixture was added to a petri dish containing cells to be transfected and then cultured the cells.

RETRACTED

### 2.4. Real-Time Quantitative Polymerase Chain Reaction (RT-qPCR)

The reverse transcription was performed to synthetize the first cDNA chain by using the PrimeScript RT Reagent Kit. Subsequently, RT-qPCR was performed using the SYBR Green qPCR mix kit (Takara, Kyoto, Japan) to quantify the relative levels of mRNAs and miRNAs. Glyceraldehyde 3-phosphate dehydrogenase (GAPDH) and U6 are used as internal references for CRABP2 and miR-579, respectively. The primers were CRABP2 Forward: 5′-CCCTGTAAGGTGAGTGCCAG-3′, Reverse: 5′- CCTGGGGTCTCCCAGAGAAT-3′; GAPDH Forward: 5′-AAGGTCGGAGTCAACGGATT-3′, Reverse: 5′-CTGGAAGATGGTGATGGGATTT-3′; miR-579 Forward: 5′-GTGCAGGGTCCGAGGT-3′, Reverse: 5′-TTAACAAAGTG CTCATAGTGC-3′; U6 Forward: 5′-CTCGCTTCGGCAGCACA-3′, and Reverse: 5′- AACGCTTCACGAATTTGCGT-3′.

### 2.5. Proliferation Assays

Cell counting kit-8 (CCK-8) assay was used to detect cell proliferation. Calu-3 cells were seeded into 96-well plates at a density of 2 × 10^3^ cells/well. Absorbance was measured at 24, 48, and 72 h after incubation with CCK-8 solutions for 2 h at 37 °C. At each time point, cells were added 10 *μ*l of 5 mg/ml CCK-8 (Keygen Biotechnology, Nanjing, China) and then incubated for 4 h. The absorbance was measured at 570 nm on the spectrophotometer.

### 2.6. Colony Formation Assay

For colony formation assays, 300 cells were seeded in 6-well plates and cultured for 12 days. PBS was utilized to wash the colonies and fixed the colonies with 4% paraformaldehyde for 30 min. Crystal violet was applied to stain the colonies with staining solution for 10 minutes, followed by the colonies which were washed with water and air-dried. Finally, the cell colonies are imaged and counted using a microscope.

### 2.7. Transwell Assay

Transwell inserts covered with Matrigel (Becton Dickinson, NJ, USA) were utilized to measure cell invasive ability. The upper chamber was added 100 *μ*l cell suspension with a density of 5 × 10^4^ cells/ml. The lower chamber was filled with 500 *μ*l medium containing 10% FBS as a chemoattractant. The cells were incubated at 37 °C for 24 h in a humidified environment with 5% CO2. A cotton swab was employed to remove the cells still on the top surface of the insert. The invade cells were fixed with methanol and stained with crystal violet at room temperature. After washed by PBS, the number of cells in five randomly fields were counted under a light microscope (Olympus Corporation, Japan).

### 2.8. Western Blotting Assay

RIPA lysis buffer (Beyotime, China) was utilized to lyse cells. The proteins were separated by electrophoresis through 10% sodium dodecyl sulfate-polyacrylamide gel electrophoresis (SDS-PAGE). The gels were followed transferred onto polyvinylidene fluoride (PVDF) membranes (MilliporeCorp, Billerica, MA, USA), and they were incubated by primary antibodies overnight in 4 °C. The primary antibodies were Anti-CRABP2 (ab211927, Abcam, Shanghai, China) and Anti-GAPDH (ab8245, Abcam, Shanghai, China). The blots was incubated for 1 h with anti-rabbit horseradish peroxidase conjugated antibody. Proteins were visualized with ECL-chemiluminescent kit (ADANTI, Wuhan, China).

RETRACTED

### 2.9. Dual-Luciferase Reporter Assay

Based on the binding site predicted by Starbase, wild-type and mutant sequences of CRABP2 were inserted into the pcDNA3.1 vector to construct CRABP2 wild-type (CRABP2-WT) and CRABP2 mutant (CRABP2-MT). Cells were co-transfected with wild-type/mutant vector and miR-579 mimic/NC using Lipofectamine 2000. Promega (Madison) dual luciferase reporter detection system was used to determine luciferase activity.

### 2.10. Statistical Analysis

Data are expressed as mean ± standard deviation (SD) from triplicate recordings. Statistical processing was carried out using SPSS and GraphPad Prism 6 software. The unpaired Student's *t*-test was used to compare date between groups that were normally distributed. *P* values less than 0.05 were considered statistically significant.

## 3. Results

### 3.1. Overexpression of miR-579 Inhibits Cell Viability and Invasion of Lung Adenocarcinoma

To detect the expressions of miR-579 in lung adenocarcinoma by using RT-qPCR, we first profiled differentially expressed genes in LUAD and corresponding paracancerous tissue samples. And we discovered that miR-579 expression was downregulated in LUAD tissues compared with corresponding paracancerous tissues (*P* < 0.05) (Figure 1(a)). Also, the expression of miR-579 was lower in LUAD cell lines H1650, A549, and Calu-3 than normal human bronchial epithelial cell line BEAS-2B (*P* < 0.05) (Figure 1(b)).

The biological function of miR-579 is determined through the gains and losses of functional experiments. MiR-579 mimic was used to overexpress miR-579 in Calu-3 cells. The transfection efficiency was measured by RT-qPCR (*P* < 0.05) (Figure 1(c)). We found that overexpression of miR-579 suppressed cell proliferation (*P* < 0.05) and colony formation ability (*P* < 0.05) (Figures 1(d) and 1(e)). In addition, overexpression of miR-579 inhibited cell invasive ability of Calu-3 cells (*P* < 0.05) (Figure 1(f)). Overall, the findings indicated that miR-579 regulated the viability and invasion of Calu-3 cells in vitro.

RETRACTED

### 3.2. Knockdown of miR-579 Promotes the Viability and Invasion of Calu-3 Cells

To further clarify the potential function of miR-579, miR-579 inhibitor was synthesized and then transfected into Calu-3 cells, and its transfection efficiency was checked. MiR-579 inhibited the expression level of miR-579 in Calu-3 cells (*P* < 0.05) (Figure 2(a)). Knockdown of miR-579 promoted cell proliferation and colony formation abilities (*P* < 0.05) (Figures 2(b) and 2(c)). In transwell experiments, knockdown of miR-579 inhibited cell invasion ability of lung adenocarcinoma (*P* < 0.05) (Figure 2(d)).

### 3.3. CRABP2 Is Regulated by miR-579

Through TargetScan, we discovered that CRABP2 was a target gene of miR-579, so we wonder whether mIR-579 affected the expression of CRABP2, and then affected the biological function of cells through CRABP2. The miR-579 binding sequences on CRABP2 mRNA were mutated from 5′-…AACCGCG…-3′ to 5′-…UUGGCGC…-3′ (Figure 3(a)). To verify that miR-579 directly target CRABP2 in Calu-3 cells, two plasmid vectors were co-transfected containing WT or MUT CRABP2 3′-untranslated regions (3'UTR) and miR-579 mimic in Calu-3 cells and then measure the luciferase activity. As we found, co-expression of miR-579 mimic and wild-type CRABP2 3'UTR could reduce luciferase activity (*P* < 0.05). In contrast, the luciferase activity had no change in Calu-3 cells that co-transfected miR-579 mimic and CRABP2 MUT 3′UTR (*P* > 0.05) (Figure 3(b)). The expression of CRABP2 was measured in LUAD cells H1650, A549 and Calu-3 and BEAS-2B. On the contrary with the expression of miR-579, we discovered that CRABP2 was overexpressed in H1650, A549, and Calu-3 cells verse BEAS-2B (*P* < 0.05) (Figure 3(c)). Also, the expression of CRABP2 was calculated after exogenous change miR-579. CRABP2 expression was reduced by overexpressing miR-579 (*P* < 0.05), and it was increased by inhibiting miR-579 in Calu-3 cells (*P* < 0.05) (Figures 3(d) and 3(e)).

### 3.4. Knockdown of CRABP2 Inhibits Cell Proliferation and Invasion of Calu-3 Cells

Si-CRABP2 was used to silence CRABP2 in Calu-3 cells, and the transfection efficiency was calculated by RT-qPCR (*P* < 0.05) and western blot (Figure 4(a)). CCK8 assay indicated that cell proliferation was suppressed when knockdown of CRABP2 in Calu-3 (*P* < 0.05) (Figure 4(b)). Cell colony formation assay displayed that knockdown CRABP2 inhibited the cell number of colony formation (*P* < 0.05) (Figure 4(c)). Transwell assay indicated that cell invasion ability was suppressed by silencing CRABP2 in Calu-3 cells (*P* < 0.05) (Figure 4(d)).

### 3.5. Overexpression of CRABP2 Reverses the Inhibition of miR-579 on Cell Proliferation and Invasion in Calu-3 Cells

CRABP2 plasmid and miR-579 mimic were co-transfected in Calu-3 cells. The RNA and protein levels of CRABP2 in Calu-3 was measured by RT-qPCR (*P* < 0.05) and western blotting (Figure 5(a)). We demonstrated that the miR-579 mimic inhibited cell proliferation, while CRABP2 overexpressed reversed the inhibition of miR-579 on cell proliferation (*P* < 0.05) (Figure 5(b)). Similarly, cell number of clone formation was found to be reduced by overexpressing miR-579, while CRABP2 inversed the reduction of miR-579 (*P* < 0.05) (Figure 5(c)). Transwell assay analysis demonstrated that miR-579 mimic suppressed invasion of Calu-3 cells, whereas CRABP2 reversed this reduction (*P* < 0.05) (Figure 5(d)). The addition of CRABP2 into Calu-3 cells could reverse the tumor suppression effects of miR-579 mimic.

RETRACTED

## 4. Discussion

Lung adenocarcinoma has a high mortality rate possibly due to delays in diagnosis due to insignificant symptoms [15]. In early LUAD, most patients are asymptomatic. Approximately 57% of lung cancers metastasize and affect the normal function of other organs and tissues [16]. Thus, the tumor biomarkers are important for early diagnosis and treatment of cancer patients.

MiRNAs are a class of small endogenous noncoding RNAs that modulate multiple human genes by mRNA degradation or repression [17]. MiRNAs can complementarily bind to the 3′-UTR of the corresponding target gene, ultimately inhibiting gene translation at transcriptional or post-transcriptional level [18]. MiR-579 has been shown to play crucial roles in biological progresses. MiR-579 is a negative prognostic factor and acts as a suppressor in melanoma [19]. MiR-579 is downregulated in squamous cell lung carcinoma and inhibits the proliferation, invasion, and migration [20]. However, the functional mechanisms of miR-579 have not been elucidated in lung adenocarcinoma. We discovered that miR-579 was low expressed in LUAD tissues and cell lines compared with corresponding paracancerous tissues and bronchial epithelial cell. MiR-579 inhibited the proliferation, colony formation, and invasion of Calu-3 cells. We also found that CRABP2 was a direct target gene of miR-579 and miR-579 regulates cell progression via targeting CRABP2 in Calu-3 cells.

CRABP2, an intracellular lipid binding protein associated with retinoic acid, is considered a key regulator of intracellular retinoic acid signaling [21]. Increasing researches indicate that CRABP2 may act as a transcription coactivator and can involve in biological behavior independent [22]. For example, CRABP2 promotes cell migration and invasion and the EMT in non-small cell lung cancer cells [23]. Consistent with the above findings, silencing of CRABP2 suppressed the proliferation, colony formation, and invasion in Calu-3 cells. On the contrary, CRABP2 acts as a suppressor factor and is related to ethnicity, nerve invasion, and postoperative treatment [24]. Similarly, CRABP2 suppresses the EMT, invasion, and metastasis of ER breast cancer cells in vitro and in vivo [25]. Therefore, we speculate that CRABP2 has tissue specificity.

RETRACTED

## 5. Conclusion

All the results indicated that the tumor suppressor function of miR-579 is exerted partly by the negative regulation of CRABP2 in LUAD. However, the specific regulatory mechanism of miR-579 remains to be further investigated. Our next work will require further investigation of the roles of miR-579/CRABP2 axis in tumorigenesis using animal model.

## Figures and Tables

**Figure 1:** Overexpression of miR-579 inhibits cell viability and invasion of lung adenocarcinoma. (a) MiR-579 expression was downregulated in LUAD tissues compared with corresponding paracancerous tissues. (b) MiR-579 expression was lower in LUAD cell lines H1650, A549, and Calu-3 than BEAS-2B. (c) MiR-579 mimic was overexpressed miR-579 in Calu-3 cells. (d) Overexpression of miR-579 suppressed cell proliferation. (e) Overexpression of miR-579 inhibited colony formation ability. (f) Overexpression of miR-579 inhibited cell invasive ability of Calu-3 cells.

**Figure 2:** Knockdown of miR-579 promotes the viability and invasion of Calu-3 cells. (a) MiR-579 inhibited the expression level of miR-579 in Calu-3 cells. (b) Knockdown of miR-579 promoted cell proliferation. (c) Knockdown of miR-579 promoted colony formation ability. (d) Knockdown of miR-579 inhibited cell invasion ability of lung adenocarcinoma.

**Figure 3:** CRABP2 was regulate by miR-579 (a) Through TargetScan, we found that CRABP2 is a direct target gene of miR-579. The miR-579 binding sequences on CRABP2 mRNA were mutated from 5′-…AACCGCG…-3′ to 5′-…UUGGCGC…-3′. (b) Co-expression of miR-579 mimic and wild-type CRABP2 3′UTR could reduce luciferase activity, and it had no change in Calu-3 cells that co-transfected miR-579 mimic and CRABP2 MUT 3′UTR. (c) CRABP2 was overexpressed in H1650, A549, and cells verse BEAS-2B. (d) The expression of CRABP2 was calculated after exogenous change miR-579. (e) CRABP2 expression was increased by inhibiting miR-579 in Calu-3 cells.

**Figure 4:** Knockdown of CRABP2 inhibits cell proliferation and invasion of Calu-3 cells. (a) Si-CRABP2 was used to silence CRABP2 in Calu-3 cells, and the transfection efficiency was calculated by RT-qPCR and western blot. (b) Cell proliferation was suppressed when knockdown of CRABP2 in Calu-3. (c) Knockdown CRABP2 inhibited cell colony formation ability. (d) Cell invasion ability was reduced by silencing CRABP2 in Calu-3 cells.

RETRACTED

**Figure 5:** MiR-579 suppresses cell proliferation and invasion by regulating CRABP2 in Calu-3 cells. (a) CRABP2 plasmid and miR-579 mimic were co-transfected in Calu-3 cells. (b) MiR-579 mimic inhibited cell proliferation, while CRABP2 overexpressed reversed the inhabitation of miR-579 on cell proliferation. (c) Clone formation was found to be reduced by overexpressing miR-579, while CRABP2 inversed the reduction of miR-579. (d) MiR-579 mimic inhibited the invasion of Calu-3 cells, while CRABP2 reversed this reduction.

## Data Availability

Data to support the findings of this study is available on reasonable request from the corresponding author.

## References

[1] Chen Z., Fillmore C. M., Hammerman P. S., Kim C. F., Wong K. K. (2014). Non-small-cell lung cancers: a heterogeneous set of diseases. *Nature Reviews. Cancer*.

[2] Miyazawa T., Marushima H., Saji H. (2019). PD-L1 expression in non-small-cell lung cancer including various adenocarcinoma subtypes. *Annals of Thoracic and Cardiovascular Surgery*.

[3] Ni M., Shi X. L., Qu Z. G., Jiang H., Chen Z. Q., Hu J. (2015). Epithelial mesenchymal transition of non-small-cell lung cancer cells A549 induced by SPHK1. *Asian Pacific Journal of Tropical Medicine*.

[4] Mollaei H., Safaralizadeh R. (2019). *MicroRNA replacement therapy in cancer.*.

[5] Lee Y. S., Dutta A. (2009). MicroRNAs in cancer. *Annual Review of Pathology*.

[6] Rupaimoole R., Slack F. J. (2017). MicroRNA therapeutics: towards a new era for the management of cancer and other diseases. *Nature Reviews. Drug Discovery*.

[7] Huang J., Weng Q., Shi Y. (2020). MicroRNA-155-5p suppresses PD-L1 expression in lung adenocarcinoma. *FEBS Open Bio*.

[8] Cao J., Geng J., Chu X., Wang R., Huang G., Chen L. (2019). miRNA-885-3p inhibits docetaxel chemoresistance in lung adenocarcinoma by downregulating Aurora A. *Oncology Reports*.

[9] Ma D. J., Zhou X. Y., Qin Y. Z., Tian Z. H., Liu H. S., Li S. Q. (2021). MiR-22-3p expression is down-regulated in lung adenocarcinoma. *Acta Biochimica Polonica*.

[10] Chen J., Zhang K., Zhi Y. (2021). Tumor-derived exosomal miR-19b-3p facilitates M2 macrophage polarization and exosomal LINC00273 secretion to promote lung adenocarcinoma metastasis via hippo pathway. *Clinical and Translational Medicine*.

[11] Li J., Zhu Z., Li S., Han Z., Meng F., Wei L. (2021). Circ_0089823 reinforces malignant behaviors of non-small cell lung cancer by acting as a sponge for microRNAs targeting SOX4^,^. *Neoplasia*.

[12] Jiao X., Liu R., Huang J. (2020). Cellular retinoic-acid binding protein 2 in solid tumor. *Current Protein & Peptide Science*.

RETRACTED

[13] Zhao H., Zhu X., Luo Y. (2021). LINC01816 promotes the migration, invasion and epithelial-mesenchymal transition of thyroid carcinoma cells by sponging miR-34c-5p and regulating CRABP2 expression levels. *Oncology Reports*.

[14] Chen Q., Tan L., Jin Z., Liu Y., Zhang Z. (2020). Downregulation of CRABP2 inhibit the tumorigenesis of hepatocellular carcinoma in vivo and in vitro.

[15] Hirsch F. R., Scagliotti G. V., Mulshine J. L. (2017). Lung cancer: current therapies and new targeted treatments. *Lancet*.

[16] Huang T. H., Wu A. T., Cheng T. S. (2019). In silico identification of thiostrepton as an inhibitor of cancer stem cell growth and an enhancer for chemotherapy in non-small-cell lung cancer. *Journal of Cellular and Molecular Medicine*.

[17] Bertoli G., Cava C., Castiglioni I. (2015). MicroRNAs: new biomarkers for diagnosis, prognosis, therapy prediction and therapeutic tools for breast cancer. *Theranostics*.

[18] Hayes J., Peruzzi P. P., Lawler S. (2014). MicroRNAs in cancer: biomarkers, functions and therapy. *Trends in Molecular Medicine*.

[19] Fattore L., Mancini R., Acunzo M. (2016). miR-579-3p controls melanoma progression and resistance to target therapy. *Proceedings of the National Academy of Sciences of the United States of America*.

[20] Wu R. R., Zhong Q., Liu H. F., Liu S. B. (2019). Role of miR-579-3p in the development of squamous cell lung carcinoma and the regulatory mechanisms. *European Review for Medical and Pharmacological Sciences*.

[21] Meng J. F., Luo M. J. (2021). CRABP2 involvement in a mechanism of Golgi stress and tumor dry matter in non-small cell lung cancer cells via ER dependent hippo pathway. *Acta Biochimica Polonica*.

[22] Wei L., Liu Y., Ma Y. (2019). C-X-C chemokine receptor 2 correlates with unfavorable prognosis and facilitates malignant cell activities via activating JAK2/STAT3 pathway in non-small cell lung cancer. *Cell Cycle*.

[23] Meng J. F., Luo M. J., Li H. B. (2021). Correlation between plasma cellular retinoic acid-binding protein 2 and proliferation, migration, and invasion of non-small-cell lung cancer cells. *Critical Reviews in Eukaryotic Gene Expression*.

[24] Li M., Li C., Lu P. (2021). Expression and function analysis of CRABP2 and FABP5, and their ratio in esophageal squamous cell carcinoma. *Open Med (Wars)*.

[25] Feng X., Zhang M., Wang B. (2019). CRABP2 regulates invasion and metastasis of breast cancer through hippo pathway dependent on ER status. *Journal of Experimental & Clinical Cancer Research*.

